The article "Sleep disturbances and PTSD: a perpetual circle?" was published in 2012. Journal: Eur J Psychotraumatol.

# Sleep disturbances and PTSD: a perpetual circle?

**DOI:** 10.3402/ejpt.v3i0.19142

**Published:** 2012-10-03

**Authors:** Saskia van Liempt

**Affiliations:** Military Mental Health, University Medical Centre, Utrecht, The Netherlands

**Keywords:** PTSD, sleep, nightmares, polysomnography, cortisol, growth hormone, memory, noradrenalin

## Abstract

**Background:**

Sleep facilitates the consolidation of fear extinction memory. Nightmares and insomnia are hallmark symptoms of posttraumatic stress disorder (PTSD), possibly interfering with fear extinction and compromising recovery. A perpetual circle may develop when sleep disturbances increase the risk for PTSD and vice versa. To date, therapeutic options for alleviating sleep disturbances in PTSD are limited.

**Methods:**

We conducted three studies to examine the relationship between sleep and posttraumatic symptoms: (1) a prospective longitudinal cohort study examining the impact of pre-deployment insomnia symptoms and nightmares on the development of PTSD; (2) a cross-sectional study examining subjective sleep measures, polysomnography, endocrinological parameters, and memory in veterans with PTSD, veterans without PTSD, and healthy controls (HCs); (3) a randomized controlled trial (RCT) (*n*=14) comparing the effect of prazosin and placebo on sleep disturbances in veterans with PTSD. In addition to these studies, we systematically reviewed the literature on treatment options for sleep disturbances in PTSD.

**Results:**

Pre-deployment nightmares predicted PTSD symptoms at 6 months post-deployment; however, insomnia symptoms did not. Furthermore, in patients with PTSD, a correlation between the apnea index and PTSD severity was observed, while obstructive sleep apnea syndrome was not more prevalent. We observed a significant increase in awakenings during sleep in patients with PTSD, which were positively correlated with adrenocorticotropic hormone (ACTH) levels, negatively correlated with growth hormone (GH) secretion, and the subjective perception of sleep depth. Also, heart rate was significantly increased in PTSD patients. Interestingly, plasma levels of GH during the night were decreased in PTSD. Furthermore, GH secretion and awakenings were independent predictors for delayed recall, which was lower in PTSD. In our RCT, prazosin was not associated with improvement of any subjective and objective sleep parameters. Only a few RCTs have been published. They show promising results for atypical antipsychotics and prazosin, the latter especially on nightmare reduction.

**Conclusions:**

Disturbed sleep due to nightmares increases the risk for PTSD. PTSD in turn leads to increased sleep fragmentation, decreased GH secretion, and frequent nightmares, which may again compromise fear extinction, synaptic plasticity, and recovery. This suggests that disturbed sleep is a precipitating and perpetuating factor in PTSD symptomatology, creating a perpetual circle. This dissertation suggests that activity of the hypothalamic–pituitary–adrenal axis and the sympathetic nervous system (SNS) is involved in disturbed sleep in patients with PTSD.

The article "Sleep disturbances and PTSD: a perpetual circle?" was published in 2012. Journal: Eur J Psychotraumatol.

This dissertation focuses on sleep in patients with a combat-related posttraumatic stress disorder (PTSD). Nightmares and insomnia are highly prevalent in patients with PTSD (Neylan et al., 1998; Ohayon & Shapiro, 2000). However, cross-sectional polysomnographic (PSG) studies on objective sleep quality in patients with PTSD leave the researchers in the field puzzled, since these studies showed only mild disturbances in objective sleep quality (Breslau et al., 2004; Hurwitz, Mahowald, Kuskowski, & Engdahl, 1998; Kobayashi, Boarts, & Delahanty, 2007; Pillar, Malhotra, & Lavie, 2000).

Sleep is important for synaptic plasticity and memory formation. Fear extinction memory is a process of “forgetting” the association between a certain neutral trigger and an aversive stimulus. Like learning, in general, fear extinction memory consolidation requires synaptic plasticity. Remarkably, sleep, and presumably rapid eye movement sleep (REMS), enhances the process of fear extinction. Longitudinal studies have reported an association between sleep disturbances in the early aftermath of trauma and the development of PTSD (Kobayashi, Sledjeski, Spoonster, Fallon, & Delahanty, 2008; Koren, Arnon, Lavie, & Klein, 2002; Mellman, Bustamante, Fins, Pigeon, & Nolan, 2002). Other studies also found that sleep disturbances before the trauma, as measured retrospectively, predicted PTSD (Bryant, Creamer, O'Donnell, Silove, & McFarlane, 2010; Mellman, David, Kulick-Bell, Hebding, & Nolan, 1995). This indicates that sleep disturbances may be related to the pathophysiology of PTSD, for instance, disruption of fear extinction memory consolidation during sleep.

Sleep may be fragmented by a number of external factors, such as sleep apneas, which lead to frequent short arousals. A high prevalence of obstructive sleep apnea syndrome (OSAS) has been reported in patients with PTSD (Krakow, Germain, et al., 2000; Krakow et al., 2004, 2006). These studies also indicated relief from PTSD when OSAS was successfully treated. When sleep is disturbed by obstructive airway events, followed by a short arousal and thus interrupted sleep, the decreased sleep quality may compromise beneficial processes during sleep and may hypothetically lead to therapy resistance or chronicity in the course of the illness.

The article "Sleep disturbances and PTSD: a perpetual circle?" was published in 2012. Journal: Eur J Psychotraumatol.

In patients with PTSD, activity of the hypothalamic–pituitary–adrenal (HPA) axis and locus coeruleus (LC)/noradrenergic system is altered, which may be responsible for overstimulation of the amygdala and related limbic structures in the brain, as well as dysregulation of the negative feedbacks system that need to dampen stress responsivity (for a review, see Sherin & Nemeroff, 2011). At night, the altered activity of these neurohormones, neurotransmitters, and limbic structures may lead to altered REMS and arousal regulation (Germain, Buysse, & Nofzinger, 2008). The alteration in stress-related biological systems may be related to insomnia and re-experiences of the trauma during REMS, when limbic structures are most active (for a review, see Dang-Vu et al., 2007). The restoration of sleep in patients with PTSD may improve sleep-dependent neuroplasticity and stimulate recovery. However, only few randomized controlled trials (RCTs) have investigated the ways to alleviate sleep disturbances in patients with PTSD. To improve sleep, the profile of sleep disturbances in patients with PTSD and the underlying neurobiological systems require further study. So far, PSG studies have not clarified regulating mechanisms involved in sleep disturbances in patients with PTSD. This warrants alternative methods for the assessment of sleep regulation in patients with PTSD.

## Research questions

This dissertation consists of several experimental studies designed to answer the following questions regarding the relationship between sleep and PTSD:

1. Do insomnia and nightmares pre-deployment predict the development of PTSD symptoms?
2. Is the prevalence of OSAS increased in patients with PTSD? Are apneas related to nightmares and insomnia complaints, or to PTSD severity?
3. Are heart rate (HR) during sleep and the nocturnal secretion of melatonin, cortisol, and ACTH altered in PTSD and is this related to decreased objective and subjective sleep quality?
4. What is the relationship between objective sleep parameters according to polysomnography and subjective sleep quality in patients with PTSD?
5. Are growth hormone (GH) secretion and memory formation disturbed by PTSD and is this due to decreased objective sleep quality?
6. What is the effect of prazosin, an α_1_-adrenoceptor antagonist, on objective and subjective sleep quality in PTSD when compared to a placebo?

## Summary of major findings

Chapter 2 shows that nightmares, but not insomnia, are associated with an increased risk of developing PTSD symptoms after military deployment. This has been studied in a sample of 453 military service members who were deployed to Afghanistan. Screening for sleep disturbances and nightmares pre-deployment may contribute to early identification of those at risk of developing PTSD symptoms.

The article "Sleep disturbances and PTSD: a perpetual circle?" was published in 2012. Journal: Eur J Psychotraumatol.

Chapter 3 shows that disturbed sleep due to obstructive apneas may exert a negative effect on PTSD symptoms as PTSD patients with OSAS have more severe PTSD complaints. Obstructive sleep apnea (OSA) is not more common in patients with PTSD compared to trauma controls (TCs) and HCs.

Chapter 4 shows that sleep is more fragmented and HR is increased in patients with PTSD compared to TCs and HCs. In this study, polysomnographic registrations and 20 min blood samples were obtained simultaneously. Plasma ACTH, cortisol, and melatonin concentrations are not significantly altered in PTSD, while a trend is seen for lower cortisol levels in the first half of the night. ACTH is positively related to the number of awakenings. Furthermore, ACTH is inversely related to the amount of slow wave sleep (SWS). Patients with PTSD exhibit a significantly decreased cortisol:ACTH ratio (CORT: ACTH) upon awakening compared to TCs. TCs demonstrate an increased CORT:ACTH during the night compared to both PTSD patients and HCs, suggesting an increased response of the adrenals upon ACTH stimulation under baseline conditions in veterans without lifetime psychiatric disorders.

Chapter 5 shows that PTSD patients have lower GH levels during the night. Fragmented sleep is inversely related to GH secretion. Noticeably, overnight memory consolidation is inversely related to awakenings. A positive relationship between memory recall and GH secretion has been observed.

Chapter 6 comprises a systematic review, showing that pharmacotherapeutic options for sleep disturbances in PTSD have not been extensively studied with RCTs. So far, best results have been described in small RCTs investigating drugs with α_1_-antagonistic properties.

Chapter 7 shows that treatment of sleep symptoms in PTSD patients with prazosin (*n*=6) has no effect on the number of awakenings or other PSG parameters and sleep diary measurements compared with placebo (*n*=6) in a small RCT. Significantly, more side effects occur after prazosin treatment.

## Repercussions of disturbed sleep

Nightmares before military deployment, that is, a period of increased risk of trauma exposure, increase the risk for PTSD symptom development in response to deployment. Furthermore, sleep apnea has been related to higher PTSD scores in PTSD patients. These observations indicate that disturbed sleep may influence PTSD symptomatology. Evidence from previous studies show that sleep promotes generalization of extinction of memory in healthy humans (Pace-Schott et al., 2009; Spoormaker et al., 2010, 2011). This indicates that disturbed sleep may directly contribute to PTSD development by means of disrupting the beneficial process of sleep with regard to fear extinction. Nightmares predominantly occur during REMS (Nielsen & Levin, 2007), while they may also occur during nonrapid eye movement sleep in PTSD patients (Hefez, Metz, & Lavie, 1987). REMS in particular seems to have an effect on fear extinction (Spoormaker et al., 2010, 2011). The observed relationship between nightmares and the risk of developing PTSD symptoms may suggest that disturbed REMS is a risk factor for PTSD.

The article "Sleep disturbances and PTSD: a perpetual circle?" was published in 2012. Journal: Eur J Psychotraumatol.

Besides, nightmares have been associated with increased noradrenalin levels (Raskind et al., 2007). Furthermore, noradrenergic activity may be involved in PTSD development (Southwick et al., 1999). Thus, alternatively, the development of PTSD and the occurrence of nightmares may be epiphenomena, both induced by increased noradrenalin levels, and may not be causally linked. Our results suggest that nightmares are a trait, making an individual more vulnerable to developing PTSD symptoms. Our study also shows that insomnia symptoms fail to predict PTSD symptoms at 6 months post-deployment when pre-deployment mood and anxiety complaints are taken into account. These results differ from the previous studies in which a positive association between the development of PTSD and insomnia symptoms before or directly after trauma exposure (Bryant et al., 2010; Koren et al., 2002; Mellman, David, et al., 1995) was observed. This may be explained by the fact that these studies did not correct for mood and anxiety complaints. The relationship between insomnia symptoms and mood and anxiety complaints is complex and may be bidirectional: insomnia symptoms may contribute to mood and anxiety complaints and—vice versa—insomnia symptoms may be moderated by mood or anxiety complaints (Abad & Guilleminault, 2005). Therefore, it is possible that mood and anxiety complaints caused by insomnia increase the risk of developing PTSD after trauma and are therefore mediators in the relation between insomnia symptoms and PTSD development. Alternatively, mood and anxiety complaints may be confounding factors, causing both insomnia symptom complaints and PTSD development. In the current design, we could not differentiate whether mood and anxiety complaints are confounding factors or mediators in the relation between insomnia symptoms and PTSD development.

OSAS was not more prevalent in patients with PTSD compared to TCs and HCs, contrary to previous uncontrolled studies that suggested indices between 60 and 90% in PTSD (Krakow, Germain, et al., 2000; Krakow et al., 2004, 2006; Yesavage et al., 2010).

The article "Sleep disturbances and PTSD: a perpetual circle?" was published in 2012. Journal: Eur J Psychotraumatol.

In these studies, screening instruments for detecting OSA may have been more sensitive than in our study, especially because some studies defined a cutoff of five events per hour. Another explanation for the high incidence of OSA in some previous studies is that the usage of benzodiazepines was not discontinued before sleep recordings, which increases the occurrence of OSA (Dolly & Block, 1982). In our study, participants with regular benzodiazepine usage were excluded, and participants with habitual benzodiazepine usage were refrained from sleep medication in the sleep laboratory. Finally, our study group consisted of middle-aged veterans, whereas other studies included either female PTSD patients or elderly veterans with PTSD. The incidence of OSA may be different in other populations with PTSD. As none of the previous studies included a control group, it cannot be concluded that the incidence of OSA is elevated in PTSD. Our study underlines the importance of controlled studies to determine whether OSA is more prevalent in PTSD than in matched controls.

Nonetheless, we did observe a positive correlation between the apnea–hypopnea index per hour and more severe PTSD. Possibly, PSTD is a risk factor for OSAS, leading to a higher incidence of OSAS in severe PTSD. Alternatively, PTSD patients who happen to suffer from OSA as well may experience symptom increases due to disturbed sleep. One uncontrolled study has suggested a positive effect on PTSD symptoms after treating OSAS with continuous positive airway pressure (Krakow, Lowry, et al., 2000). Possibly, when sleep is important for recovery, and is compromised by arousals due to obstructive events, OSAS may intervene with response to treatment. It would be advisable to screen for OSAS in case of snoring and other indicators of OSAS, especially in therapy resistant patients.

In this dissertation, we also report a putative working mechanism for how sleep disturbances may influence daytime complaints. We found that GH levels during the night were decreased in PTSD patients, compared to HCs. Reduced GH secretion correlated with awakenings during the night. A regression analyses with delayed recall as dependent showed that both sleep fragmentation and GH secretion were significant predictors for memory retention of a declarative memory task. This indicated that sleep-dependent memory consolidation is disturbed in PTSD due to decreased nocturnal GH secretion and more interrupted sleep. More research is warranted to confirm these novel findings.

GH receptors are present in the hippocampus (Lai, Emtner, Roos, & Nyberg, 1991). It is suggested that GH stimulates neuroplasticity in the hippocampus (Kim, Grover, Bertolotti, & Green, 2010). A recent functional MRI study in healthy volunteers showed decreased hippocampus activation and decreased performance on a memory task after a night of experimentally induced sleep fragmentation (Van der Werf et al., 2009). Thus, sleep fragmentation can have an effect on hippocampal function. In patients with PTSD, structural and functional changes in the hippocampus also have been reported (Bremner, 2006). Interestingly, insomnia complaints in PTSD are inversely related to volume on the CA3 area of the hippocampus (Neylan et al., 2010). Decreased GH secretion may hypothetically be related to decreased hippocampus activity and possibly also hippocampal volume in PTSD. The effect of GH on neurons of the hippocampus during sleep deprivation has been shown in a recent preclinical study (Kim et al., 2010). This study shows that in the absence of GH during sleep deprivation *N*-methyl-d-aspartate (NMDA) receptor-mediated synaptic currents decreased in hippocampal neurons. Moreover, NMDA receptor loss was observed, as was a decline in long-term potentiation. These processes normalized when GH injections were administered during sleep deprivation. Reduced GH secretion may possibly be related to decreased hippocampal functioning in patients with PTSD. The relationship between treatment response to a selective serotonin reuptake inhibitor (SSRI) and neurogenesis in the hippocampus was reported in a preclinical study (Santarelli et al., 2003). In combat-related PTSD, a relationship between treatment response and hippocampal volume has also been suggested (Vermetten, Vythilingam, Southwick, Charney, & Bremner, 2003). Future research should indicate whether GH secretion is related to hippocampus volume or functioning in PTSD. Furthermore, the relationship between hippocampal volume, neurogenesis, and treatment response remains to be elucidated.

The article "Sleep disturbances and PTSD: a perpetual circle?" was published in 2012. Journal: Eur J Psychotraumatol.

## Characteristics of sleep disturbances in patients with PTSD

Sleep in PTSD patients was characterized by more awakenings compared to TCs and HCs. Increased awakenings were also reported in earlier studies (Breslau et al., 2004; Habukawa, Uchimura, Maeda, Kotorii, & Maeda, 2007; Mellman, Kulick-Bell, Ashlock, & Nolan, 1995). In agreement with a meta-analysis of PSG studies in PTSD total sleep time (TST) in our study was unchanged, as was REMS (Kobayashi et al., 2007). Our study did not demonstrate reduced SWS, which was decreased according to the meta-analysis on PSG studies in PTSD (Kobayashi et al., 2007).

In our study, cortisol levels tended to be lower during the first half of the night in patients with PTSD. ACTH levels were not elevated, which may have been due to the sample sizes (effect size *f*=0.42, required total sample 58). Both cortisol and ACTH levels were correlated with SWS, while in a regression analysis only ACTH was an independent predictor for SWS. Interestingly, ACTH levels also correlated positively with the number of awakenings. ACTH secretion is stimulated by CRH activity. The correlation between ACTH and both SWS and awakenings may therefore be indicative for CRH being involved in waking and SWS regulation in PTSD. CRH is known to inhibit SWS and increase awakening during sleep (Steiger, 2007). It was previously observed that CRH is increased in cerebrospinal fluid and plasma in PTSD patients (Baker et al., 1999). Furthermore, in a meta-analysis on PSG studies, SWS was decreased in patients with PTSD. Further explorations of CRH in sleep complaints in PTSD may in time contribute to the development of novel treatment strategies.

We also hypothesized increased activity of the LC in PTSD-related sleep fragmentation. The LC is a nucleus in the pons where noradrenergic neuronal cell bodies are located, which have projections throughout the brain. Also the sympathetic nervous system (SNS) is innervated by the LC. Noradrenergic activity stimulates awakening by stimulating the ascending reticular arousal system (ARAS) and inhibiting sleep-promoting ventrolateral preoptic nucleus (VLPO) activity (Saper, Scammell, & Lu, 2005). Noradrenaline is therefore one of the key players in the so-called “sleep/wake switch,” a system involving the ARAS, VLPO, and related neurotransmitters (Saper et al., 2005). We did indeed find increased HR in PTSD patients in comparison with TCs and HCs, which is in accordance with previous work and indicative for increased sympathetic activity (Muraoka, Carlson, & Chemtob, 1998; Woodward et al., 2009). We did not find any relationships between HR and awakenings in patients with PTSD or in the combined sample. This may have been due to the small sample size; only eight PTSD patients were allowed to enter the analyses after excluding those with cardiovascular medication, which was used by a relative large portion of the PTSD patients (3/13). Recent research has indeed shown increased cardiovascular risk in patients with PTSD (Boscarino, 2012). Possibly, the elevated SNS activity during the night may increase the risk of developing cardiovascular complications in PTSD.

The involvement of noradrenaline in PTSD-related sleep disturbances was further supported by RCTs that demonstrate a positive effect of prazosin on nightmares and insomnia in PTSD (Germain et al., 2012; Raskind et al., 2003, 2007; Taylor et al., 2008).

In summary, HRs were significantly higher during sleep in PTSD patients, indicating increased SNS activity. Furthermore, we found that awakenings were increased in patients with PTSD. Interestingly, awakenings were positively related to ACTH secretion. In addition, perceived sleep quality was inversely related to the number of awakenings. Therefore, it is advised to calculate the number of awakenings in future PSG studies, as this seems to be a robust alteration in objective sleep quality in PTSD.

The article "Sleep disturbances and PTSD: a perpetual circle?" was published in 2012. Journal: Eur J Psychotraumatol.

## Treatment of sleep disturbances in PTSD

Insomnia and nightmares are frequently residual complaints in PTSD after successful psychotherapy with cognitive behavior therapy (Zayfert & De Viva, 2004) or pharmacotherapy with SSRIs (Davidson, Rothbaum, Van der Kolk, Sikes, & Farfel, 2001). In Chapter 5, we systematically reviewed studies that were published before 2006, investigating pharmacotherapeutic options for sleep disturbances in patients with PTSD. Our review shows that even though benzodiazepines are the most widely prescribed sleep medication, their effects on sleep disturbances in PTSD have not been extensively studied by RCTs. Only two small RCTs (*n*=6, *n*=22), with short treatment periods of 1 week, have been conducted (Cates, Bishop, Davis, Lowe, & Woolley, 2004; Mellman, Bustamante, David, & Fins, 2002). Several small RCTs have indicated that prazosin is superior to placebo in improving subjective sleep in patients with PTSD (Germain et al., 2012; Raskind et al., 2003, 2007; Taylor et al., 2008). Also, RCTs have shown the efficacy of the atypical antipsychotics olanzapine and risperidone as add-on therapy alongside an SSRI (Rothbaum et al., 2008; Stein, Kline, & Matloff, 2002). Prazosin and quetiapine, another atypical antipsychotic, were similar in their short-term effects (Byers, Allison, Wendel, & Lee, 2010). However, quetiapine more often led to discontinuation due to adverse side effects. RCTs showed that guanfacine, an α_2_-adrenoceptor agonist, was not effective in treating nightmares and insomnia (Neylan et al., 2006).

Objective measurements of sleep were employed in two studies. One RCT investigating the effect of prazosin estimated REMS and TST with an eye tracker (Taylor et al., 2008). This study suggested increased TST and REMS after prazosin treatment. Another RCT with three groups (prazosin, placebo, and a cognitive behavior therapy) measured polysomnography, the golden standard for measuring sleep architecture (Germain et al., 2012). In this study, no differences over time were seen between groups on all PSG parameters and most subjective sleep measures. Only the number of reported nightmares was reduced in the active treatment groups in comparison with placebo. We also measured polysomnography and sleep questionnaires in a small RCT on the effect of prazosin, as has been described in Chapter 6. Our study was in agreement with the observations from the study by Germain et al. (2012) that PSG parameters, Pittsburgh sleep quality index scores, and sleep diary measurements did not differ between groups. We also measured the number of awakenings pre- and posttreatment but did not find a significant difference. This may have been due to the intensity of our study.

The article "Sleep disturbances and PTSD: a perpetual circle?" was published in 2012. Journal: Eur J Psychotraumatol.

A meta-analysis including all RCTs on prazosin using polysomnography should be performed to further analyze the effect of prazosin on objective sleep quality in PTSD. However, polysomnography may not be a suitable method for detecting the underlying mechanism of nightmares in PTSD. Alternative methods may further elucidate the suggested effect of blocking α_1_-adrenoceptor activity on nightmares. For instance, functional MRI with combined EEG during sleep may demonstrate decreased activity of limbic brain structures during (REM) sleep in relation to a reduction in nightmare complaints.

In summary, prazosin and atypical antipsychotics are effective in the treatment of PTSD-related sleep complaints. However, prazosin does not increase the risk of a metabolic syndrome and has therefore a more favorable side effect profile. One RCT showed that sleep-focused behavioral therapy was as effective as prazosin on both insomnia and nightmares. Imaginary rehearsal therapy (IRT) is also effective for those suffering from nightmares, but cannot be applied in those without dream content recall. Prazosin treatment, IRT, and sleep-focused cognitive behavior therapy (CBT) are all effective for treating sleep disturbances (Germain et al., 2012; Krakow et al., 2001). Unfortunately, prazosin is no longer available in the Netherlands. Distribution has been stopped because prazosin was not regularly prescribed to patients suffering from hypertension and benign prostate hypertrophy. Alternatively, quetiapine, or the selective α_1_-adrenoceptor antagonists doxazosin and alfuzosine, may be useful. However, RCT is warranted to assess the efficacy of doxazosin and alfuzosine in PTSD-related sleep disturbances. Also sleep-focused psychotherapy may not always be available to PTSD patients, as not all psychologists and psychiatrists are familiar with these interventions. The choice of treatment depends on the preference of the patient and availability of therapeutic options.

## The HPA-axis and adaptation after trauma exposure

Changes in the functioning of the HPA axis have repeatedly been associated with PTSD (for a review, see de Kloet et al., 2006). Generally, increased responsivity to dexamethasone has been reported. Also, increased CRH levels have been demonstrated in cerebrospinal fluid and plasma (Baker et al., 1999; de Kloet et al., 2008). Results on peripheral cortisol values are inconsistent. Most studies report low or normal cortisol concentrations compared with controls (Klaassens, Giltay, Cuijpers, van Veen, & Zitman, 2012; Meewisse, Reitsma, de Vries, Gersons, & Olff, 2007). A previous study suggests that HPA-axis alterations after traumatic stress are also related to trauma exposure and not merely with PTSD symptoms (de Kloet, Vermetten, Bikker, et al., 2007; de Kloet, Vermetten, Heijnen, et al., 2007). We therefore included two control groups in our study: one group that comprised veterans without lifetime psychiatric disorder and one control group of nondeployed–or otherwise traumatized—individuals. ACTH values in our study did not differ at night or in the morning between the three groups. Cortisol levels tended to be lower in PTSD during the first half of the night. However, significant group differences in the ratio of CORT:ACTH were demonstrated. The CORT:ACTH ratio reflects the responsiveness of the adrenals upon ACTH stimulation. It appeared to be a sensitive measure for changes in HPA axis activity. It is advisable to test not only plasma cortisol in future research but also, if possible, to measure ACTH levels in order to calculate the ratio of CORT:ACTH.

The article "Sleep disturbances and PTSD: a perpetual circle?" was published in 2012. Journal: Eur J Psychotraumatol.

In our small study, with a limited power to detect significant differences, we were able to demonstrate group differences in CORT:ACTH ratio. First, an increased CORT:ACTH ratio was observed in TCs during the night compared with both PSTD patients and HCs. This alteration in TCs compared with both PTSD patients and HCs was first described by Golier et al. (2007) in Gulf War veterans. Second, in PTSD patients a decreased CORT:ACTH ratio was observed upon awakening. Both observations may be ascribed to the responsiveness of the adrenals upon ACTH stimulation. Hyporesponsive adrenals to ACTH may explain the decreased ratio in PTSD patients. In contrast, in TCs higher responsive adrenals to ACTH may explain the observed difference. We postulate that adaptation to trauma exposure leads to more responsive adrenals to ACTH, while a reduced responsiveness of the adrenals upon ACTH stimulation is seen in those who do not accomplish adaptation. This may implicate insufficient cortisol levels to induce an adequate inhibiting feedback response to HPA-axis activity in PTSD. In contrast, in TCs higher cortisol secretion may induce a more rapid normalization of a stress response, which may be reflected by “resilience” and adaptation.

Noticeably, glucocorticoid receptors (GR) are hyperresponsive in PTSD patients, who demonstrate exaggerated responses to dexamethasone administration (de Kloet, Vermetten, Heijnen et al., 2007; Rohleder, Joksimovic, Wolf, & Kirschbaum, 2004; Yehuda, Halligan, Golier, Grossman, & Bierer, 2004). A higher number of GR has also been reported before exposure to potentially traumatic events, in service members who developed PTSD symptoms post-deployment (Van Zuiden et al., 2011). It is unknown whether in patients with PTSD the reduced response of the adrenals to ACTH stimulation and elevated GR number and responsivity may be related. Presumably, low responsiveness of the adrenals to ACTH may imply relatively lower cortisol levels upon stimulation, and, subsequently, an upregulation of GR receptors as a compensatory mechanism. One study also found elevated sensitivity of the GR receptor in TCs compared with HCs (de Kloet, Vermetten, Heijnen, et al., 2007). When cortisol secretion is increased in TCs after ACTH stimulation, and GR receptor enhancement takes place after trauma, the HPA-axis may be even further sensitized for the negative feedback response of cortisol in TCs.

The article "Sleep disturbances and PTSD: a perpetual circle?" was published in 2012. Journal: Eur J Psychotraumatol.

Future research investigating stress and posttraumatic symptoms should focus on the dynamic characteristics of the HPA-axis, for instance, calculating CORT:ACTH ratios. In addition, sensitivity and upregulation of receptors involved in the HPA-axis should be further explored.

## Concluding remarks and recommendations

Sleep has been studied with polysomnography in the early days of PTSD research. However, the lack of objective findings in PSG studies urged the need to develop alternatives for measuring sleep in patients with PTSD. This dissertation shows that sleep in patients with PTSD is characterized by frequent awakenings at night, according to polysomnographic registrations. The number of awakenings in patients with PTSD is associated with HPA-axis functioning, subjectively perceived sleep, and, interestingly, GH secretion and memory consolidation. Furthermore, this dissertation supports the idea that disturbed sleep exerts a negative effect on PTSD symptomatology. First, nightmares before military deployment predicted PTSD symptom development, independently early life trauma, mood, and anxiety symptoms. Second, a positive correlation was observed between PTSD severity and the number of sleep apneas, which may indicate an increase in PTSD symptoms when sleep quality is compromised by external factors. Our results suggest that disturbed sleep increases the risk for PTSD. PTSD, in turn, leads to increased sleep fragmentation, decreased GH secretion, and frequent nightmares, which may again compromise fear extinction, synaptic plasticity, and recovery. This suggests that disturbed sleep is a precipitating and perpetuating factor in PTSD symptomatology, possibly creating a perpetual circle.

The article "Sleep disturbances and PTSD: a perpetual circle?" was published in 2012. Journal: Eur J Psychotraumatol.

Longitudinal studies are warranted to investigate whether the differences in sleep fragmentation, GH secretion, and increased HR during sleep, found in our cross-sectional studies, are “trait or state” phenomena. In addition, more research is needed to further investigate the effects of sleep disruptions on fear extinction memory consolidation. New approaches are advised, such as combined functional MRI/EEG studies to elucidate brain activation patterns and functional connectivity during sleep. More studies investigating sleep-dependent neuroplasticity and growth factors during sleep are also needed to further explore whether sleep disturbances affect biological underpinnings of psychiatric disease and recovery through the effect of sleep on synaptic plasticity.
